# Blockade of leukocyte haptokinesis and haptotaxis by ketoprofen, diclofenac and SC-560

**DOI:** 10.1186/1471-2172-12-64

**Published:** 2011-11-12

**Authors:** Saulius Paskauskas, Audrius Parseliunas, Vachtang Kerkadze, Rainer Nobiling, Jan Schmidt, Eduard Ryschich

**Affiliations:** 1 Department of Surgery, University of Heidelberg, Heidelberg, Germany; 2 Institute of Physiology, University of Heidelberg, Heidelberg, Germany; 3 University of Health Sciences, Kaunas, Lithuania

## Abstract

**Background:**

Nonsteroidal anti-inflammatory drugs (NSAID) represent a one of the most widely used anti-inflammatory substances. Their anti-inflammatory effects are mainly based on inhibition of cyclooxygenase. The potential direct effect of NSAID on leukocyte migration was poorly investigated. Using time-lapse microscopy and 96-well fluorescence-based assay, we studied the effect of three different NSAID, ketoprofen, diclofenac and SC-560, on leukocyte haptokinesis and haptotaxis in vivo and in vitro.

**Results:**

NSAID induced an immediate inhibiting effect on leukocyte migration both in vitro and in vivo. This effect was dose-dependent and was not restricted to a specific type of leukocytes. The inhibition of leukocyte migration by NSAID was partially re-stored after removal of inhibiting agent. Only complete blockade of leukocyte migration was accompanied by a strong reduction of [Ca^2+^]i.

**Conclusions:**

NSAID strongly supress leukocyte migration. The results of the present study may have important clinical implications since blockade of leukocyte migration can be achieved after topical application of NSAID.

## Background

Migration is an important feature of leukocytes which represents a pre-requisite for normal leukocyte function in physiological processes such as protection against infection or foreign antigens. Under pathological conditions, leukocytes infiltrate tissue which locally produces pro-inflammatory substances and chemokines. This process is known as leukocyte recruitment. The normal ability for active movement is an important pre-requisite for the effective recruitment of leukocytes from the microvascular circulation [1]. The blockade of leukocyte migration can abrogate the process of leukocyte recruitment and inflammation. Therefore, the modulation of leukocyte migration has been proposed as a potential therapeutic approach for the treatment of several inflammatory diseases such as psoriasis, eczema, multiple sclerosis and arthritis [2,3].

Dependent on the tissue structure, two types of non-directed leukocyte migration can be identified: two- and three-dimensional haptokinesis. Two-dimensional leukocyte haptokinesis can be found on two-dimensional surfaces, such as inner vessel walls, the peritoneum and the pleura. Three-dimensional haptokinetic migration occurs in the tissue which contains cellular or fibrillar extracellular matrix components promoting leukocyte movement [1]. Prevailing random haptokinetic leukocyte migration becomes directional (hapto- or chemotactic), if a gradient of chemotacic agent is present in the tissue. Chemotaxis is induced by soluble, freely diffusing compounds that lead to preferential signaling and actin-rich protrusions at the leading edge. In contrast to chemotaxis, haptotaxis represents the directed migration toward chemoattractants which are immobilized on tissue structures, such as interstitial collagens or stromal cell network [1].

Nonsteroidal anti-inflammatory drugs (NSAID) are one of the most widely used anti-inflammatory substances. The major anti-inflammatory effect of NSAID is the inhibition of cyclooxygenase (COX) enzyme system which blocks prostaglandin synthesis and leads in consequence, to reduction of inflammation, pain and fever [4]. It has also been shown that COX inhibition by NSAID reduces migratory activity of leukocytes which therefore leads to a reduction of leukocyte recruitment into the inflamed tissue. Although the effect of some NSAID such as aspirin, indometacin or ketoprofen on leukocyte migration was investigated in several previous studies [5,6], these studies were mainly focused on the changes of migration of polymorphonucelar leukocytes (PMNs) and did not analyze effects of NSAID at the single leukocyte level. In the present study, we studied the effect of three different NSAID, ketoprofen, diclofenac and SC-560 on the haptokinesis and haptotaxis of PMNs and activated lymphocytes at the single cell level in vitro and in vivo using time-lapse microscopy. The study was in particular aimed to identify the effective concentrations of NSAID which can suppress leukocyte migration. Furthermore, the toxic potential of these NSAID and the role of Ca^2+ ^were analyzed. Ketoprofen and diclofenac are known to inhibit both COX-1 and COX-2 whereas SC-560 belongs to the group of COX-1-selective inhibitors.

## Methods

### Leukocytes preparation

Polymorphonuclear leukocytes (PMNs) or lymphocytes were isolated from human venous peripheral blood using density gradient centrifugation (Biocoll, Biochrom AG, Berlin, Germany). Microscopic examination showed that at least 90% of isolated polymorphonuclear leukocytes were represented by neutrophils. For the 3D haptotaxis, isolated human PMNs or lymphocytes were used immediately after isolation. In some experiments, lymphocytes were activated for 5 days at 37°C using 1.5 μg/ml of concanavalin A (Calbiochem, Darmstadt, Germany) in Iscove's Modified DMEM supplemented with 10% FCS (c.c.pro, Oberdorla, Germany). To study inhibitory effects on leukocyte migration, the following NSAID were used: ketoprofen (ct-Arzneimittel GmbH, Berlin, Germany), diclofenac (Novartis Pharma GmbH, Nürnberg, Germany), SC-560 (Cayman Chemical, Ann Arbor, Michigan, USA).

### Analysis of leukocyte haptokinesis

Leukocyte migration in collagen matrix in vitro was analyzed using modified 96-wells collagen matrix assay as previously described [7]. For this assay, 100 μl/well of collagen mixture was prepared and polymerized for 30 min at 37°C. 100 μl of leukocyte suspension (10.000 cells/well) containing different concentrations of NSAID was layered upon the collagen gel. Plates were incubated at 37°C for 60 Min to allow migrating leukocytes to invade into collagen gel. The suspension of non-invading leukocytes were washed using Multi-Reagent Washer (Dynatech, Gaithersberg, USA). 5 μM/well of Calcein AM (MoBiTec, Goetingen, Germany) were added and incubated for 30 min. The fluorescence was measured using multilable counter (Victor 1420, Perkin&Elmer Wallac GmbH, Freiburg, Germany). The number of invaded leukocytes was calculated using reference concentration of leukocytes and was expressed as a percentage of migrating leukocytes to total leukocyte number.

For time-lapse microscopy, 4 × 10^5 ^cells in 50 μl of PBS were added to the collagen mixture in a petri plate prior the polymerization. Digital time-lapse microscopy was performed after application of different concentrations of ketoprofen to the gel as previously described [7]. Leukocyte movement was recorded for 20 min. Subsequently, gel preparation was washed with PBS and recorded for further 30 min. Six experiments for each group were performed.

### Analysis of leukocyte haptotaxis

Leukocytes invasion into the collagen matrix was analyzed. For this aim, 5 μl of collagen matrix mixture were prepared on ice as previously described [7]. Additionally, this mixture contained IL-8 (10 ng/ml) or SDF-1 (100 ng/ml; R&D Systems, Wiesbaden, Germany) and ketoprofen and filled into the glass square tube (1 × 1 mm, Vitrocom, Mountain Lakes, NJ, USA). Collagen matrix was allowed to polymerize for 30 min at 37°C. 5 μl of leukocyte suspension (2.000 cells/μl) was added upon collagen matrix. The tube was fixed in the upright position and incubated at 37°C for 3 hours for neutrophils or 24 hours for lymphocytes. The distance of leukocyte invasion into the matrix was recorded using microscope and measured using Histo software (W. Gross, University of Heidelberg, Germany).

### Intravital microscopy

Five male lysEGFP-ki mice (10-12 weeks) were used. These mice allow an excellent visualization of EGFP-expressing neutrophils using fluorescence microscopy. To induce local leukocyte activation and extravasation, 20 μl of IL-8 (R&D Systems) was injected onto the auricle. An excessive amount of ketoprofen gel (2.5% ketoprofen; Effekton, Teofarma, Pavia, Italy) was applied on the skin of the auricle before or 60 min after IL-8 injection. Blood vessels were visualized using intravenous injection of 0.6 mg of TRITC-labelled albumin (Sigma Aldrich, Deisenhofen, Germany). Time-lapse intravital microscopy of auricle was performed using fluorescence microscope (Axio Observer, Zeiss GmbH, Jena, Germany) combined with image deconvolution (Huygens Essential, SVI, Hilversum, Netherlands). The speed and the fraction of migrating leukocytes were measured using Capimage software (Version 5.02, Zeintl GmbH, Heidelberg, Germany). All experiments were approved by the local committee of animal care (Regierungspräsidium Karlsruhe).

### Toxicity assays

Potential cytotoxic effect of NSAID on PMNs was measured using Calcein AM assay (MoBiTec) as described in manufacturer's instruction. In brief, leukocytes were incubated with different concentrations of NSAID for 60 min at 37°C and loaded with 5 μM Calcein AM. Vital cells metabolised calcein and produced fluorescent signal which was measured using fluorimeter (Victor 1420) and expressed as a percent of the non-treated control. Three experiments for every substance were performed.

### [Ca^2+^]i measurement

Ca^2+ ^was measured as previously described by Nobiling and Bührle [8]. In brief, isolated leukocytes were incubated in collagen gel for 30 min and were loaded with 2 μM of FURA-2 AM (Molecular Probes, Eugene, USA). Intracellular Ca^2+ ^([Ca^2+^]i) signal was recorded at alternately 340 and 360 nm wavelength for 15 sec at three stages: at baseline, after application of 2 and 4 mM ketoprofen and after removal of ketoprofen by washing. [Ca^2+^]i concentration was calculated as 340/360 nm ratio and expressed in μM.

### Statistical analysis

Statistical analysis was performed using SPSS software (Version 11.5.1, SPSS Inc., Chicago, USA). All data are given as mean ± SD. To study differences between the groups, Wilcoxon or Mann-Whitney-U-test were used, if appropriate. p < 0.05 was considered as significant.

## Results

### NSAID inhibit leukocyte migration in vitro

The influence of different concentrations of NSAID on leukocyte haptokinesis in collagen matrix was studied using a 96-well Calcein assay. Neutrophils or activated lymphocytes showed an active migration in the collagen matrix. There were no inhibiting effects on leukocyte migration of low concentrations of NSAID. We found that all used NSAID (ketoprofen, diclofenac, SC-560) inhibited migration of both neutrophils and lymphocytes in a dose-dependent manner in vitro (Figure 1A-C). Depending on the selecting drug and on the leukocyte population (PMNs or lymphocytes), the dose of 0.6-4.0 mM led to complete blockade of leukocyte migration (Figure 1). Ketoprofen showed the highest IC50 on leukocyte migration whereas diclofenac had the lowest IC50 (Table 1).

**Table 1:** Mean IC50 (μM) for inhibition of leukocyte migration by NSAID.

substance	PMNs	lymphocytes
ketoprofen	760	1050
diclofenac	110	70
SC-560	200	220

**Figure 1:** **A-C: Effect of NSAID on leukocyte migration: changes of migratory activity of isolated human lymphocytes and granulocytes were measured using 96-wells calcein AM assay**. Ketoprofen (A), diclofenac (B) or SC-560 (C) showed a dose-dependent inhibition of PMNs and lymphocyte migration. **D-F: **Toxic effect of NSAID on PMNs: Leukocytes were incubated for 60 min with different concentrations of ketoprofen (D), diclofenac (E) and SC-560 (F). Cell number was measured using Calcein AM uptake. Only highest concentrations of ketoprofen (4 mM) and diclofenac (2.5-5 mM) induced significant reduction of the leukocyte number.

Toxicity assay showed that only highest concentrations of ketoprofen (4 mM) and diclofenac (2.5-5 mM) led to significant reduction of the cell number. 5 mM diclofenac destroyed almost all leukocytes after 60 min incubation (Figure 1D-E). No reduction of leukocyte number was found after incubation with SC-560.

### Inhibition of leukocyte migration by NSAID is reversible

Since all NSAID showed a similar inhibiting effect on leukocyte migration, further experiments using time-lapse microscopy were focused on the effects of ketoprofen. We found that the percent of migrating leukocytes in collagen gel was 87 ± 6%, whereas the mean speed of leukocyte migration was 3.2 ± 1.3 μm/min. Migrating leukocytes showed a multipolar polarized shape and stable random movement (haptokinesis) over a long time period.

Leukocyte migration in control group was stable (Figure 2). The concentration of 0.08 mM ketoprofen significantly decreased speed, whereas a concentration of 4 mM caused a total blockade of leukocyte migration (Figure 2). These effects were found immediately after application of NSAID. Washing-out of ketoprofen led to a recovery of leukocyte migration, although the speed of movement after recovery did not achieve its baseline value (Figure 2C-D).

**Figure 2:** **Effect of ketoprofen on single leukocyte migration: A-B: Leukocyte migration was studied using digital time-lapse microscopy**. Ketoprofen caused a dose-dependent inhibition of leukocyte speed (A) which partially recovered after the removal of ketoprofen (B). **C: **Representative images of migrating leukocytes in collagen matrix at baseline, leukocyte depolarization 5 min after application of 2 mM of ketoprofen and partial restitution of leukocyte migration after removal of ketoprofen. **D-E: **Blockade of activated leukocytes using topic application of ketoprofen in vivo: quantitative analysis of leukocyte speed (**D**) and representative image of intravital microscopy (**E**). Application of ketoprofen gel 60 min after IL-8 injection caused a rapid leukocyte depolarization and movement stop (leukocytes are showed as green-fluorescent cells).

### NSAID blocked leukocytes invasion in vitro and prevented leukocyte recruitment in vivo

To study leukocyte haptotaxis, we analyzed leukocyte invasion into the collagen matrix with or without chemokine. In this assay, leukocytes showed a superficial invasion into the collagen matrix, if no chemoattractants were added to the collagen. IL-8 or SDF-1 induced a strong directed invasion of both neutrophils and lymphocytes into the collagen matrix (Figure 3A-B). Interestingly, addition of 0.4 and 2 mM ketoprofen to the matrix inhibited leukocyte penetration in a dose-dependent manner whereas 4 mM ketoprofen prevented leukocyte invasion into the matrix (Figure 3A-B).

**Figure 3:** **Leukocyte repulsion by ketoprofen: Representative images (A) and quantitative analysis (B) of leukocyte penetration of collagen matrix in vitro**. **C: **Prevention of leukocyte infiltration after topic application of ketoprofen in vivo prior the IL-8 injection. **D: **Representative image of intravital microscopy. Leukocytes appeared in green, blood vessels were visualized using i.v. injection of TRITC-conjugated albumin (orange). IL-8 strongly activated leukocyte extravasation and migration, whereas almost no leukocytes were found if ketoprofen gel was locally applied on skin prior the IL-8 injection.

Intravital microscopy showed that the cutaneous injection of IL-8 induced a strong intravascular activation and extravasation of leukocytes, which infiltrated cutaneous tissue within several minutes (Figure 3C-D, Additional file 1, Movie 1). Interestingly, the local application of ketoprofen gel to the auricle led to the lost of leukocyte polarization and the blockade of leukocyte migration (Figure 2D-E), which was observed within several minutes after ketoprofen application. If ketoprofen gel was applied before IL-8 injection, leukocyte recruitment and infiltration were almost absent (Figure 3C-D, Additional file 2, Movie 2).

### Ketoprofen decreases intracellular [Ca^2+^]_i _in migrating human granulocytes in vitro

Leukocytes of control experiments showed a well-polarised shape and a constant [Ca^2+^]_i _signal. Ketoprofen concentration of 2-4 mM caused a rapid leukocyte depolarisation (Figure 2C). No significant changes of [Ca^2+^]_i _were found after addition of 2 mM ketoprofen (Figure 4). Interestingly, the increase of ketoprofen concentration to 4 mM led to a dramatic decrease of [Ca^2+^]i signal. The higher the initial value of [Ca^2+^]_i_, the sharper was its decline (Figure 4). The washing-out of ketoprofen led to a partial restoration of [Ca^2+^]i signal (Figure 4).

**Figure 4:** **Individual values of [Ca^2+^]i changes (A) and the time-course of a single representative measurement (B)**. [Ca^2+^]i was measured using cell labelling with Fura-2 and ultrasensitive single-cell-based fluorimetry. 4 mM, but not 2 mM ketoprofen caused rapid decrease of [Ca^2+^]i, which was partially restored after removal of ketoprofen.

## Discussion

In the present study, the effect of three different NSAID, ketoprofen, diclofenac, SC-560 on leukocyte haptotaxis and haptokinesis was analyzed. We found that all used NSAID inhibited leukocyte migration of in a dose-dependent manner both in vivo and in vitro. At the single cell level, NSAID inhibited both leukocyte speed and the fraction of migrating leukocytes. This effect occurred immediately after NSAID application and was partially restored after removal of inhibiting agent. Interestingly, inhibiting effect of NSAID was not dependent on the type of leukocytes, since migration of both PMNs and lymphocytes was inhibited by equivalent concentrations. The inhibitory effect of ketoprofen was reproducible in Calcein-based assay and in time-lapse microscopy. Interestingly, inhibiting effect of NSAID on leukocyte migration is reversible. As shown in the present study, leukocytes re-store their migration if NSAID concentration decreases. Results of the present study correspond well with previous results which analyzed the effect of some NSAID such as aspirin, indomethacin or ketoprofen on leukocyte migration [5,6]. These studies showed that NSAID inhibit chemotaxis of polymorphonuclear leukocytes (PMNs). In contrast to previous studies, we analyzed both PMN and T cell migration, studied haptotactic movement and showed changes of leukocyte migration at the single cell level in vivo and in vitro.

We also showed that 4 mM ketoprofen stopped leukocyte invasion into the IL-8 or SDF-1-containing matrix in vitro. This effect was also studied in vivo using time-lapse intravital microscopy. IL-8 and SDF-1 are two important chemokines which control leukocyte chemo- and haptotaxis by binding to the CXCL8 and to CXCL12 chemokine receptor, respectively [9,10]. Leukocyte recruitment and infiltration were effectively prevented if ketoprofen was locally applied in vivo prior the pro-inflammatory stimulation. We believe that the repellent action of NSAID is the direct consequence of their blocking effect on leukocyte migration both in vivo and in vitro. Ketoprofen blocked leukocyte migration for at least one hours. The potential resuming of leukocyte movement after the longer exposure to ketoprofen were not analyzed.

Previous studies showed that NSAID inhibit COX at a concentration of 10^-5^-10^-3^M. The inhibition of COX is a major, but not a single mechanism of potential NSAID effects. In the present study, the initial inhibition of leukocyte migration was found at NSAID concentrations beginning from 10-50 μM and the IC50 varied from 70 to 1050 μM. This concentrations is 10-fold higher than the highest known IC50 required for COX inhibition for diclofenac and SC-560 whereas this difference for ketoprofen is 500-fold [11,12]. Therefore, we believe that the direct inhibition of leukocyte migration through NSAID cannot only represent a COX-dependent phenomenon, but other mechanisms may participate in the NSAID action on leukocyte migration. The data of the present study correspond well with results of previous studies. These studies demonstrated that NSAID have an inhibiting effect on chemotaxis of PMNs at high concentrations in vitro which was independent of their potency as prostaglandin inhibitors [6,13]. In contrast to these studies, we showed that not only chemotactic, but also haptokinetic migratory activity of single leukocytes can be blocked by NSAID. Furthermore, almost all previous studies focused on the changes of migration of polymorphonuclear leukocytes, whereas the effect of NSAID on lymphocyte migration was poorly investigated. Results of the present study demonstrated that NSAID have similar inhibiting effects on migration of both PMNs and lymphocytes and that lymphocyte movement can be stopped by NSAID.

Other previous studies showed that low concentrations of NSAID inhibit COX production by activated mast cells and macrophages and reduce inflammation-induced leukocyte infiltration [14,15]. Although COX inhibition by low concentrations of NSAID can reduce leukocyte infiltration in inflamed tissue, this effect can be produced by rather different mechanism than the direct inhibition of leukocyte migration. We believe that COX-related effects of NSAID are not a major factor for the direct inhibition of leukocyte migration. Furthermore, we propose that other possible mechanisms of NSAID action such as inhibition of intracellular ATP [16,17], calcium metabolism [18] or [Ca^2+^]i-dependent myosin II activation [19,20] can be responsible for the inhibition of leukocyte migration. The results of the present study confirmed the important role of Ca^2+ ^signaling in NSAID action and showed that the stop of leukocyte migration by ketoprofen was accompanied by the dramatic decrease of [Ca^2+^]i and by the cytotoxic effect whereas partial inhibition of leukocyte migration did not cause a significant reduction of [Ca^2+^]i and did not induce cell toxicity.

Concentrations of NSAID, which are required for blockade of leukocyte migration, are high. As showed in previous studies, high NSAID concentration cause toxic side effects, if these substances are systemically applied [21]. However, NSAID do not induce systemic toxic side effects after topic application as gel or salve formulation [22,23] or after intraarticular injection. Previous studies showed that ketoprofen has a high percutaneous penetration [24,25]. The present study showed that the topic application of concentrated ketoprofen gel (2.5% ketoprofen) rapidly blocked migration of cutaneous leukocytes. We believe that the suppression of leukocyte migration can represent one of the pharmacological effects of NSAID after the topic application in clinical use.

It is known that other anti-inflammatory drugs such as dexamethasone suppress leukocyte migration [26]. It binds to its intracellular receptor and inhibits gene expression by binding to negative regulatory promoter regions or through protein/protein interactions [26]. The effect of NSAID corresponds well with effect of dexamethasone. As shown in the present study, ketoprofen can block SDF-1 and IL-8-mediated leukocyte migration. In accordance with our results, previous studies demonstrated that dexamethasone augmented intracellular chemokine signaling and inhibited SDF-1-induced chemotaxis of resting T cells [27]. Furthermore, dexamethasone also suppressed IL-8-induced chemotaxis of PMN through inhibition of endogenous chemokine production [28]. It can be proposed that inhibition of endogenous chemokine production by ketoprofen or other NSAID can also participate in the inhibition of leukocyte migration.

## Conclusions

In summary, our results demonstrate that ketoprofen, diclofenac and SC-560 have a direct suppressive effect on haptotaxis and haptokinesis of polymorphonuclear leukocytes and lymphocytes. This effect is dose-dependent and partially reversible after removal of inhibiting agent. This process is probably induced by COX-dependent and COX-independent mechanisms whereas complete blockade, but not the partial inhibition of migration is accompanied by changes of Ca^2+^signaling. These results indicate a possible discrete mechanism of NSAID action which may be identified in further experiments. The findings of the present study may have an important clinical implications since the blockade of leukocyte migration can also be expected after local application of NSAID in humans.

## Authors' contributions

SP: most experiments in vitro, manuscript preparation; AP and VK: design and data analysis of leukocyte migration experiments in vitro; RN: design, control and data aquisition of Ca^2+ ^measurement, JS: data analysis, preparation of the manuscript; ER: idea and concept, study design, haptotaxis experiments, intravital microscopy, manuscript preparation. All authors read and approved the final manuscript.

## Supplementary Material

Additional file 1 **Time-lapse intravital microscopy of leukocyte extravasation in mouse cutaneous tissue (auricle)**. Cutaneous inflammation was induced by injection of IL-8. Neutrophils express EGFP and appear in green. Blood vessels are labelled using intravenous injection of TRITC-labelled albumin. Real-time recording of 30 min was compressed to time-lapse sequence of 7 sec. control experiment; IL-8 induces an immediate extravasation and migration of leukocytes from the venule. Click here for file

Additional file 2 **Time-lapse intravital microscopy of leukocyte extravasation in mouse cutaneous tissue (auricle)**. Cutaneous inflammation was induced by injection of IL-8. Neutrophils express EGFP and appear in green. Blood vessels are labelled using intravenous injection of TRITC-labelled albumin. Real-time recording of 30 min was compressed to time-lapse sequence of 7 sec. Application of ketoprofen gel prior injection of IL-8 blocks intravascular leukocyte adhesion and extravasation. Click here for file
